The article "The generation and characterization of novel Col1a1FRT-Cre-ER-T2-FRT and Col1a1FRT-STOP-FRT-Cre-ER-T2 mice for sequential mutagenesis" was retracted in 2016. Reasons: errors in the results or conclusions; unreliable results or conclusions.

# The generation and characterization of novel *Col1a1^FRT-Cre-ER-T2-FRT^* and *Col1a1^FRT-STOP-FRT-Cre-ER-T2^* mice for sequential mutagenesis

**DOI:** 10.1242/dmm.021204

**Published:** 2015-09-01

**Authors:** Minsi Zhang, David G. Kirsch

**Affiliations:** 1 Department of Pharmacology and Cancer Biology, Duke University, Durham, NC 27708, USA; 2 Department of Radiation Oncology, Duke University Medical Center, Box 91006, LSRC Bldg, Rm B230, Durham, NC 27708, USA

**Keywords:** Mouse models, Sequential mutagenesis, Dual recombinase technology

## Abstract

Novel genetically engineered mouse models using the Cre-*loxP* or the Flp-*FRT* systems have generated useful reagents to manipulate the mouse genome in a temporally-regulated and tissue-specific manner. By incorporating a constitutive Cre driver line into a mouse model in which *FRT*-regulated genes in other cell types are regulated by Flp-*FRT* recombinase, gene expression can be manipulated simultaneously in separate tissue compartments. This application of dual recombinase technology can be used to dissect the role of stromal cells in tumor development and cancer therapy. Generating mice in which Cre-ER^T2^ is expressed under Flp-*FRT*-mediated regulation would enable step-wise manipulation of the mouse genome using dual recombinase technology. Such next-generation mouse models would enable sequential mutagenesis to better model cancer and define genes required for tumor maintenance. Here, we generated novel genetically engineered mice that activate or delete Cre-ER^T2^ in response to Flp recombinase. To potentially utilize the large number of Cre-*loxP*-regulated transgenic alleles that have already been targeted into the *Rosa26* locus, such as different reporters and mutant genes, we targeted the two novel Cre-ER^T2^ alleles into the endogenous *Col1a1* locus for ubiquitous expression. In the *Col1a1^FRT-Cre-ER-T2-FRT^* mice, Flp deletes Cre-ER^T2^, so that Cre-ER^T2^ is only expressed in cells that have never expressed Flp. In contrast, in the *Col1a1^FRT-STOP-FRT-Cre-ER-T2^* mice, Flp removes the STOP cassette to allow Cre-ER^T2^ expression so that Cre-ER^T2^ is only expressed in cells that previously expressed Flp. These two new novel mouse strains will be complementary to each other and will enable the exploration of complex biological questions in development, normal tissue homeostasis and cancer.

## Abstract (precis)

**Summary:** We generated two mouse strains expressing Cre-ER^T2^ under Flp*-FRT* regulation. These tools enable sequential mutagenesis in the same or different cells to study development, tissue homeostasis and diseases such as cancer.

## INTRODUCTION

Genetically engineered mouse models are ideal for studying complex mammalian biological processes *in vivo*. Advances in genetic engineering have enabled the development of increasingly more precise, controlled manipulation of the mouse genome so that more intricate biological questions can be explored. Site-specific recombinase systems, such as the Cre-*loxP* and the Flp-*FRT* systems, were developed to allow for temporally-regulated and tissue-specific gene modification (Dymecki, 1996; O'Gorman et al., 1991; Orban et al., 1992; Sauer and Henderson, 1988). A large number of conditional mouse alleles utilizing the Cre-*loxP* system have been generated. These include various *loxP*-flanked genes and a number of endogenous-promoter-driven Cre-recombinase alleles that are constitutively expressed. Cre recombinase expressed from endogenous promoters enables tissue-specific deletion of DNA flanked by *loxP* sites to alter gene expression. The resulting tissue-specificity for recombination of the *loxP* sites decreases the likelihood of embryonic lethality. For example, *Villin-Cre* (El Marjou et al., 2004), which is expressed in the entire intestinal and colonic epithelium, and *Fapbl^4X@-132^-Cre* (Saam and Gordon, 1999), which is expressed in the distal two thirds of the small intestine and the entire colonic epithelium, can be used to express the embryonically lethal oncogenic KRAS^G12D^ by recombining *Kras^loxP-STOP-loxP-G12D^* (Jackson et al., 2001) to generate diffuse colonic hyperplasia in mice (Haigis et al., 2008). However, gene modification in the embryo might not fully recapitulate gene manipulation in the adult to model somatic gene mutations that lead to the development of sporadic cancers. One way to circumvent this limitation is to exogenously deliver Cre recombinase to the adult mice via infection with replicative-deficient adenoviruses (Adeno-Cre) (Wang et al., 1996). For example, intratracheal delivery of Adeno-Cre to adult mice with *Rb^FL/FL^* and *p53^FL/FL^* mutations (Marino et al., 2000) generated primarily small cell lung tumors that closely resembled human small cell lung cancer (Meuwissen et al., 2003). In addition to small cell lung tumors, this method also generated lung adenocarcinomas as well as medullary thyroid carcinomas both in mice that also developed small cell lung tumors and in mice that did not. This drawback to using viral vectors, particularly in cancer biology, is due to the fact that many cell types can be infected by the adenovirus. Thus, the cancer-initiating cell (i.e. cell of origin) can vary between tumors from different animals as well as different tumors within the same animal. This heterogeneity might lead to phenotypic differences in these mouse models of cancer. To further limit the expression of Cre to specific cell types within an organ, Cre can be expressed from the adenovirus using a cell-type-specific promoter (Sutherland et al., 2011, 2014).

The article "The generation and characterization of novel Col1a1FRT-Cre-ER-T2-FRT and Col1a1FRT-STOP-FRT-Cre-ER-T2 mice for sequential mutagenesis" was retracted in 2016. Reasons: errors in the results or conclusions; unreliable results or conclusions.

Innovations in site-specific recombinase systems continue to improve tissue specificity and temporal regulation of gene expressions. For example, fusion proteins consisting of Cre recombinase and a mutated estrogen receptor that preferentially binds to the metabolites of the estrogen analog tamoxifen, such as Cre-ER^T2^, have been generated (Indra et al., 1999). These fusion proteins allow for tamoxifen-inducible Cre recombinase to translocate into the nucleus and modify the genome. These Cre-fusion proteins allow temporal activation of oncogenes and/or deletion of tumor suppressor genes in the adult mouse in a cell-type-specific manner to generate cancer (Blum et al., 2013).

**RESOURCE IMPACT**

**Background**

The Cre-*loxP* and, more recently, the Flp-*FRT* recombinase systems are widely used to generate transgenic mouse models to study a variety of human diseases, including cancer. One major drawback of these tools is that, for each of the individual systems, the genetic mutations are generated at the same time, which limits the scope of questions that can be explored. Multiple recombinase systems can be combined to better temporally and spatially restrict gene mutations in *in vivo* models.

**Results**

To develop a Cre-*loxP* and Flp*-FRT* dual recombinase system that allows for more controlled manipulation of the mouse genome, the authors used Cre-ER^T2^, a fusion protein that allows for tamoxifen-inducible and temporal gene manipulation. Cre-ER^T2^ was inserted into the endogenous *Col1a1* locus to generate *Col1a1^FRT-Cre-ER-T2-FRT^* and *Col1a1^FRT-STOP-FRT-Cre-ER-T2^* mice. The *Col1a1* locus was chosen so that *Rosa26*, a locus used for constitutive, ubiquitous gene expression in mice, could be used for the expression of other genes. The authors showed that Cre-ER^T2^ is widely expressed in a variety of tissues: a single injection of intraperitoneal tamoxifen in *Col1a1^FRT-Cre-ER-T2-FRT^; Rosa26^mTmG/+^* mice efficiently deleted tdTomato and expressed eGFP via the *Rosa26^mTmG^* fluorescent reporter. Furthermore, the authors validated the *Col1a1^FRT-STOP-FRT-Cre-ER-T2^* allele in an autochthonous tumor model by crossing this allele to *Kras^FRT-STOP-FRT-G12D/+^; p53^FRT/FRT^; Rosa26^mTmG/+^* mice. The authors showed that, after tumor initiation, local or systemic injections of 4-hydroxytamoxifen in these mice can induce Cre-ER^T2^-mediated recombination of the *Rosa26^mTmG^* allele to generate eGFP-positive tumor parenchyma or stroma in a Flp-*FRT*-regulated manner.

The article "The generation and characterization of novel Col1a1FRT-Cre-ER-T2-FRT and Col1a1FRT-STOP-FRT-Cre-ER-T2 mice for sequential mutagenesis" was retracted in 2016. Reasons: errors in the results or conclusions; unreliable results or conclusions.

**Implications and future directions**

These two new mouse models, in which the Flp-*FRT* system regulates the expression of Cre-ER^T2^, can be used in combination with other *FRT-* and *loxP*-regulated alleles, as well as tissue-specific Flp or viral Flp delivery, to introduce different mutations over time in the same or different cells to study development, tissue homeostasis and diseases such as cancer. For example, these strains will be valuable tools to study sequential mutagenesis in cancer progression and the roles of genes in mediating tumor maintenance and response to therapy.

Recently, a second site-specific recombination system, Flp-*FRT*, which originated from *Saccharomyces* *cerevisiae*, has been applied to study cancer. Similar to Cre, Flp recombinase recognizes 34-bp sequences of DNA termed *FRT* sites. Like *Kras^loxP-STOP-loxP-G12D^* mice, investigators have generated mice in which *Kras^G12D^* is regulated by a transcriptional terminator sequence flanked by *FRT* sites in the endogenous promoter (*Kras^FRT-STOP-FRT-G12D^*) (Young et al., 2011). Similar to *p53^FL^* mice, we previously generated mice with the DNA-binding domain of p53 flanked by *FRT* sites (*p53^FRT^*) (Lee et al., 2012). When the *p53^FRT^* alleles are combined with *Kras^FRT-STOP-FRT-G12D^* mice, Flp can generate primary sarcomas, lung cancer and pancreatic cancer (Lee et al., 2012; Moding et al., 2015, 2014; Schönhuber et al., 2014).

The use of only one recombinase system to mutate multiple genes limits the scope of cancer research because all genetic manipulations are completed at the same time. In the case of mutations that drive cancer, the use of a single recombinase system prohibits the study of sequential mutagenesis to determine how the order of different driver gene mutations affects tumor phenotypes. Moreover, the consequence of a gene mutation at tumor initiation could be different from a mutation that is acquired later during tumor development. Indeed, when a single recombinase system is used to mutate multiple genes simultaneously, it is possible that cells might adapt to the loss of a gene at tumor initiation in ways that are different than if the same gene had been mutated later during tumor development. This might be particularly important for genetic experiments designed to identify therapeutic targets that are required for cancer maintenance because, in certain cases, inhibition of a target at the time of cancer initiation might lead to a different outcome than when a target is inhibited in an established tumor.

Others have demonstrated that the Flp-*FRT* and the Cre-*loxP* systems can be used sequentially. For example, lung adenocarcinoma has been generated by sequentially delivering Flp recombinase by adenovirus and Cre recombinase either by adenovirus or by tamoxifen to activate Cre-ER in mice harboring *Braf^FRT-STOP-FRT-V600E^* and either *p53^FL/FL^* or *Cdkn2a^FL/FL^* mutations (Shai et al., 2015). Likewise, pancreatic adenocarcinoma has been generated by sequential mutagenesis, where first *Kras^FRT-STOP-FRT-G12D^* and *Rosa26^FRT-STOP-FRT-Cre-ER-T2^* are recombined by *Pdx1-Flp* to generate pancreatic tumors harboring oncogenic KRAS and the Cre-ER^T2^ fusion protein, then tamoxifen is delivered to the animal to activate Cre-ER^T2^ to recombine *p53^FL/FL^* in the pancreatic tumors, resulting in pancreatic tumors with both KRAS and p53 mutations (Schönhuber et al., 2014).

The article "The generation and characterization of novel Col1a1FRT-Cre-ER-T2-FRT and Col1a1FRT-STOP-FRT-Cre-ER-T2 mice for sequential mutagenesis" was retracted in 2016. Reasons: errors in the results or conclusions; unreliable results or conclusions.

Here, we generated novel genetically engineered mice that activate or delete Cre-ER^T2^ in response to Flp recombinase. Specifically, we generated two new mouse strains in which Cre-ER^T2^ is knocked into the endogenous *Col1a1* locus so that the *Rosa26* locus can be used for other genes or reporters of interest. In one allele, *Col1a1^FRT-Cre-ER-T2-FRT^*, Cre-ER^T2^ is flanked by *FRT* sites. In the other allele, *Col1a1^FRT-STOP-FRT-Cre-ER-T2^*, Cre-ER^T2^ is regulated by a *FRT*-STOP-*FRT* cassette. In *Col1a1^FRT-Cre-ER-T2-FRT^* mice, cells will only express Cre-ER^T2^ and have the capacity for tamoxifen-mediated recombination of *loxP* sites if they have never had prior exposure to Flp recombinase. Therefore, this strain will be useful for studying genes in stromal cells of established tumors that are initiated by Flp. In contrast, in *Col1a1^FRT-STOP-FRT-Cre-ER-T2^* mice, in which Cre-ER^T2^ is downstream from a *FRT*-STOP-*FRT* cassette, cells will only express Cre-ER^T2^ and have the capacity for tamoxifen-mediated recombination of *loxP* sites after Flp-mediated removal of the STOP cassette. Therefore, this strain will be useful for sequential mutagenesis within tumor cells or for modifying the tumor cell genome in established cancers. Thus, these two new mouse strains will be complementary to each other and will enable the exploration of complex biological questions in cancer, normal development and tissue homeostasis.

## RESULTS

### Generation of Flp-*FRT*-regulated Cre-ER^T2^ alleles

In order to develop technology for sequential mutagenesis *in vivo* using two site-specific recombinase systems, we generated *Col1a1^FRT-Cre-ER-T2-FRT^* and *Col1a1^FRT-STOP-FRT-Cre-ER-T2^* mice. The rationale to generate *Col1a1^FRT-Cre-ER-T2-FRT^* mice was to enable whole animal ubiquitous expression of Cre-ER^T2^ until exposure to Flp recombinase (Fig. 1A). After Flp-mediated recombination of the *FRT* sites, cells are no longer able to express Cre-ER^T2^ and therefore lose the ability to delete DNA flanked by *loxP* sites following exposure to tamoxifen. In this way, different mutations can be introduced in adjacent cells *in vivo* so that the consequences for intercellular interactions, such as those between cancer cells and stromal cells, can be studied. The rationale to generate *Col1a1^FRT-STOP-FRT-Cre-ER-T2^* was that initially no cell expresses Cre-ER^T2^ because transcription of Cre-ER^T2^ is terminated by an upstream *FRT*-site-flanked transcription STOP cassette (Fig. 1B). However, after Flp-mediated recombination, the STOP cassette is excised. Therefore, these cells can initiate transcription of the Cre-ER^T2^ fusion protein, which, in response to subsequent exposure to tamoxifen, translocates into the nucleus to recombine DNA flanked by *loxP* sites. Cells without exposure to Flp will not be able to undergo Cre-mediated DNA recombination. In this way, the *Col1a1^FRT-STOP-FRT-Cre-ER-T2^* allele enables sequential mutations within the same cell over time. First, one mutation occurs in the cell from Flp recombinase, and then tamoxifen activates Cre recombinase in the same cell to mutate a second gene to study how the order of gene mutations affects cellular outcome. In addition, multiple genes might be mutated by Flp recombinase to initiate tumor development. Then, the role of a *loxP*-flanked gene in tumor maintenance can be studied because only the tumor cell will express Cre-ER^T2^. This allele can therefore be used to identify potential therapeutic targets.

The article "The generation and characterization of novel Col1a1FRT-Cre-ER-T2-FRT and Col1a1FRT-STOP-FRT-Cre-ER-T2 mice for sequential mutagenesis" was retracted in 2016. Reasons: errors in the results or conclusions; unreliable results or conclusions.

**Fig. 1.** **Sequential mutagenesis with Flp and Cre recombinases in *Col1a1^FRT-Cre-ER-T2-FRT^* and in *Col1a1^FRT-STOP-FRT-Cre-ER-T2^* mice.** (A) *Col1a1^FRT-Cre-ER-T2-FRT^* mice will express Cre-ER^T2^ recombinase ubiquitously from the *Col1a1* locus. Exposure to Flp leads to excision of the Cre-ER^T2^ coding sequence flanked by *FRT* sites in the same cell and terminates Cre recombinase expression. Any other DNA flanked by *FRT* sites will be excised at the same time. Therefore, in these cells, subsequent tamoxifen exposure does not lead to Cre-mediated recombination of *loxP* sites. Without prior exposure to Flp, tamoxifen leads to Cre-ER^T2^ translocation into the nucleus and excision of *loxP* sites. (B) *Col1a1^FRT-STOP-FRT-Cre-ER-T2^* mice do not express Cre-ER^T2^ at baseline. Cells exposed to Flp undergo excision of *FRT* sites including the STOP cassette upstream of Cre-ER^T2^, which results in transcription of Cre-ER^T2^. Subsequent tamoxifen exposure then leads to Cre-mediated recombination of *loxP* sites specifically in these cells. Cells without prior exposure to Flp do not recombine *loxP* sites when exposed to tamoxifen.

The article "The generation and characterization of novel Col1a1FRT-Cre-ER-T2-FRT and Col1a1FRT-STOP-FRT-Cre-ER-T2 mice for sequential mutagenesis" was retracted in 2016. Reasons: errors in the results or conclusions; unreliable results or conclusions.

To generate mice in which the expression of Cre-ER^T2^ is regulated by the Flp-*FRT* recombinase system and to fully utilize the large number of Cre-*loxP*-regulated transgenic alleles in the *Rosa26* locus, such as fluorescent reporters and mutant genes, the two novel Cre-ER^T2^ alleles were targeted into the endogenous *Col1a1* locus for ubiquitous expression (Fig. 2A,B). Targeting constructs for the generation of *Col1a1^FRT-Cre-ER-T2-FRT^* and *Col1a1^FRT-STOP-FRT-Cre-ER-T2^* mice consisted of the sequence from the *Col1a1* genomic DNA, CAG promoter, Cre-ER^T2^ regulated by *FRT* sites, and a neomycin selection cassette flanked by *attP* and *attB* sites. Therefore, transcription of the targeted Cre-ER^T2^ recombinase will be driven from the endogenous *Col1a1* locus and enhanced by the addition of a CAG promoter. Constructs of the two Cre-ER^T2^ alleles were electroporated into 129/SVJae embryonic stem (ES) cells and successfully targeted ES cells were selected by neomycin (G418) treatment. Positively selected ES cells were analyzed for successful homologous recombination by Southern blot of genomic DNA (Fig. 2C,D). Correctly targeted ES clones were injected into C57BL/6 blastocysts and male high-percentage chimeras were selected to breed with C57BL/6 females to identify germline transmission of the Cre-ER^T2^ alleles. The neomycin selection cassettes were removed by PhiC31-integrase-mediated recombination of the *attP* and *attB* sites *in vivo* by crossing the mice to the pre-existing *Rosa26^PhiC31^* strain (Raymond and Soriano, 2007).

**Fig. 2.** **Schematics for *Col1a1*-directed expression of *FRT-Cre-ER^T2^-FRT* and *FRT-STOP-FRT-Cre-ER^T2^*, the removal of the neomycin selection cassette, and Southern blot for successful homologous recombination.** Schematic of the *Col1a1^FRT-Cre-ER-T2-FRT^* (A) and *Col1a1^FRT-STOP-FRT-Cre-ER-T2^* (B) alleles. The neomycin cassette is used for selection of ES cells with integration of the targeting construct. PhiC31 integrase is used to remove the neomycin selection cassette *in vivo* after germline transmission. Locations of genotyping primers are indicated on each schematic. (C) Southern blot analysis indicates successful homologous recombination of the *Col1a1^FRT-Cre-ER-T2-FRT-NEO^* allele in the E2, E1 and B7 clones. The B7 clone was used to generate the *Col1a1^FRT-Cre-ER-T2-FRT-NEO^* line. (D) Southern blot analysis indicates successful homologous recombination of the *Col1a1^FRT-STOP-FRT-Cre-ER-T2-NEO^* allele in the E1, C1 and B11 clones. The B11 clone was used to generate the *Col1a1^FRT-STOP-FRT-Cre-ER-T2-NEO^* line.

The article "The generation and characterization of novel Col1a1FRT-Cre-ER-T2-FRT and Col1a1FRT-STOP-FRT-Cre-ER-T2 mice for sequential mutagenesis" was retracted in 2016. Reasons: errors in the results or conclusions; unreliable results or conclusions.

Germline transmission of *Col1a1^FRT-Cre-ER-T2-FRT-NEO^* was verified by PCR for the construct-specific neomycin selection cassette on tail-tip DNA (Fig. 3A). Heterozygosity for the knock-in allele was demonstrated by PCR for the wild-type *Col1a1* locus (Fig. 3A). Successful PhiC31-mediated excision of the neomycin selection cassette was verified by PCR for gene products specific to the recombined neomycin selection cassette (excised NEO), the unrecombined neomycin selection cassette (NEO), the wild-type *Col1a1* locus and the mutant *PhiC31* allele (Fig. 3B).

**Fig. 3.** **Germline transmission, and successful PhiC- and FlpO-mediated recombination of *attB/attP* and *FRT* sites.** (A) PCR of tail DNA for the neomycin cassette of the *Col1a1^FRT-Cre-ER-T2-FRT-NEO^* and wild-type *Col1a1* locus indicate germline transmission of a single copy of the *Col1a1^FRT-Cre-ER-T2-FRT-NEO^*allele. (B) PCR for the recombined neomycin cassette (excised NEO), unrecombined neomycin cassette (NEO), wild-type *Col1a1* locus and mutant PhiC31 allele indicate successful PhiC31-mediated deletion of the neomycin selection cassette in the *Col1a1^FRT-Cre-ER-T2-FRT-NEO^* allele, generating the *Col1a1^FRT-Cre-ER-T2-FRT^* allele. (C) PCR of tail DNA for the neomycin cassette of the *Col1a1^FR^^T-STOP-FRT-Cre-ER-T2-NEO^* and wild-type *Col1a1* locus indicate germline transmission of a single copy of the *Col1a1^FRT-STOP-FRT-Cre-ER-T2-NEO^* allele. (D) PCR for the recombined neomycin cassette (excised NEO), unrecombined neomycin cassette (NEO), presence of STOP cassette, wild-type *Col1a1* locus and mutant PhiC31 allele indicate successful PhiC31-mediated deletion of the neomycin selection cassette in the *Col1a1^FRT-STOP-FRT-Cre-ER-T2-NEO^* allele, generating the *Col1a1^FRT-STOP-FRT-Cre-ER-T2^* allele. Note that the amplified PCR product of the excised NEO band for the *Col1a1^FRT-Cre-ER-T2-FRT^*allele is slightly larger than that of the *Col1a1^FRT-STOP-FRT-Cre-ER-T2^* allele owing to the presence of the *FRT* site in between the FWD1 and REV1 primers (see Fig. 2 for schematics with the location of the *FRT* sites relative to the primers).

Germline transmission of a single copy of *Col1a1^FRT-STOP-FRT-Cre-ER-T2-NEO^* was verified by PCR for the construct-specific STOP cassette, the neomycin selection cassette and the wild-type *Col1a1* locus on tail-tip DNA (Fig. 3C). Deletion of the neomycin selection cassette by PhiC31 was verified by PCR for gene products specific for the recombined neomycin selection cassette (excised NEO), the unrecombined neomycin selection cassette (NEO), the STOP cassette, the wild-type *Col1a1* locus and the mutant *PhiC31* allele (Fig. 3D). One founder mouse for each of the novel Cre-ER^T2^ strains was used to propagate the colony.

The article "The generation and characterization of novel Col1a1FRT-Cre-ER-T2-FRT and Col1a1FRT-STOP-FRT-Cre-ER-T2 mice for sequential mutagenesis" was retracted in 2016. Reasons: errors in the results or conclusions; unreliable results or conclusions.

### Characterization of Flp-*FRT*-regulated Cre-ER^T2^ mice

To examine Cre-mediated recombination at a cellular level, tissues from *Col1a1^FRT-Cre-ER-T2-FRT^; Rosa26^mTmG/+^* mice were examined by immunofluorescence with and without tamoxifen treatment (Fig. 4). Without Cre-mediated recombination, the *Rosa26^mTmG^* allele transcribes only the tdTomato fluorescent protein. After Cre-mediated excision of tdTomato, eGFP is expressed from the same locus. Because these mice are heterozygous for the *Rosa26^mTmG^* allele, any expression of eGFP indicates Cre-mediated excision of tdTomato. In tissues taken from 6-week-old mice (*n*=2) without tamoxifen treatment (Fig. 4A), expression of tdTomato was widespread, and there was minimal tissue-specific eGFP expression. Tissues with some eGFP expression included the pancreas (Fig. 4Avii) and, to a lesser extent, a few skeletal muscle fibers (Fig. 4Aiii). When tissues from 6-month-old mice (*n*=3) obtained 30 days after treatment with a single dose of 75 mg tamoxifen/kg body weight in corn oil by intraperitoneal injection were examined (Fig. 4B), there was widespread eGFP expression and minimal tdTomato retention. The tissue with highest tdTomato retention was the brain (Fig. 4Bxxxii), where there was diffuse low tdTomato expression and regions of high eGFP expression (Fig. 4Bxxxi). This might reflect diffusion limitations of tamoxifen metabolites across the blood-brain barrier, or brain-specific expression from the *Col1a1* locus, synthesis of functional eGFP protein and degradation of tdTomato. The lower expression of tdTomato in the brain tissue of *Col1a1^FRT-Cre-ER-T2-FRT^; Rosa26^mTmG/+^* mice treated with tamoxifen as compared to untreated controls (Fig. 4Axxxii) suggests that the rate of degradation of tdTomato plays a greater role. Additionally, it seems that certain cell types do have higher tdTomato or higher eGFP expression than others, which could be due to the activity of the *Rosa26* locus or perhaps a consequence of the way the tissue is affected by processing. For example, the endothelial cells of the brain (Fig. 4Axxxii) have higher tdTomato expression than the neurons. The glomeruli of the kidney (Fig. 4Axx) have higher tdTomato expression than the collecting ducts. Overall, the lung parenchyma seems to have lower tdTomato expression (Fig. 4Axii) than other tissues such as the brain (Fig. 4Axxxii).

**Fig. 4.** **Characterization of tamoxifen-mediated Cre-ER^T2^ activity in *Col1a1^FRT-Cre-ER-T2-FRT^* mice.** (A) Immunofluorescence of tissues from 6-week-old *Col1a1^FRT-Cre-ER-T2-FRT^; Rosa26^mTmG/+^* mice (*n*=2) without tamoxifen treatment show widespread tdTomato with tissue-specific minimal to no eGFP expression, with the pancreas showing the most Cre-ER^T2^ leakiness (Avii). (B) Immunofluorescence of tissues collected 30 days after one dose of intraperitoneal tamoxifen in 6-month-old mice (*n*=3) show extensive Cre-mediated expression of eGFP and tissue-specific tdTomato degradation. Note that the brain (Bxxxii) has the highest amount of tdTomato retention as well as areas of low/no eGFP expression. Scale bars: 50 µm.

The article "The generation and characterization of novel Col1a1FRT-Cre-ER-T2-FRT and Col1a1FRT-STOP-FRT-Cre-ER-T2 mice for sequential mutagenesis" was retracted in 2016. Reasons: errors in the results or conclusions; unreliable results or conclusions.

To determine the activity of Cre-ER^T2^ in *Col1a1^FRT-Cre-ER-T2-FRT^; Rosa26^mTmG/+^* mice in the absence of tamoxifen, tissues from 4-month-old (*n*=2) and 6-month-old (*n*=3) mice without tamoxifen treatment were examined (Fig. 5). The tissues with the most widespread eGFP expression without tamoxifen treatment in the 6-month-old mice include the pancreas (Fig. 5Bvii), the liver (Fig. 5Bxv) and the skeletal muscle (Fig. 5Biii). There was a time-dependent tissue-specific increase in eGFP expression when comparing the 4-month-old and 6-month-old mice (Fig. 5A,B). For example, the skeletal muscle fibers in the 4-month-old mice (Fig. 5Aiii) had less eGFP expression than those in the 6-month-old mice (Fig. 5Biii). Additionally, the pancreas of the 4-month-old mice (Fig. 5Avii) had less eGFP expression than the pancreas of the 6-month-old mice (Fig. 5Bvii). The liver of both the 4-month-old (Fig. 5Axv) and the 6-month-old (Fig. 5Bxv) mice had similar eGFP expression. In contrast, the brain had no eGFP expression with the exception of a subset of the vasculature in both the 4-month-old mice (Fig. 5Axxxi) and the 6-month-old mice (Fig. 5Bxxxi). Taken together, these results demonstrate that there is time-dependent and tissue-specific Cre-ER^T2^ activity in *Col1a1^FRT-Cre-ER-T2-FRT^* mice in the absence of tamoxifen, with the brain tissue being the least affected organ, and the pancreas, liver and skeletal muscle fibers being the most affected organs. In addition, tamoxifen potently induces Cre-ER^T2^-mediated recombination of unrecombined *loxP* sites.

**Fig. 5.** **Characterization of tamoxifen-independent Cre-ER^T2^ activity in *Col1a1^FRT-Cre-ER-T2-FRT^* mice.** (A) Immunofluorescence of tissues from 4-month-old *Col1a1^FRT-Cre-ER-T2-FRT^; Rosa26^mTmG/+^* mice (*n*=2) without tamoxifen treatment show time- and tissue-dependent leakiness of Cre-ER^T2^, with more widespread eGFP expression in the skeletal muscle (Aiii), pancreas (Avii) and liver (Axv). (B) Immunofluorescence of tissues from 6-month-old *Col1a1^FRT-Cre-ER-T2-FRT^; Rosa26^mTmG/+^* mice (*n*=3) without tamoxifen treatment show increased time- and tissue-dependent leakiness of Cre-ER^T2^, with more widespread eGFP expression in the skeletal muscle (Biii), pancreas (Bvii) and liver (Bxv). The skeletal muscle and the pancreas show the most apparent increase in eGFP expression from 4 to 6 months. Scale bars: 50 µm.

The article "The generation and characterization of novel Col1a1FRT-Cre-ER-T2-FRT and Col1a1FRT-STOP-FRT-Cre-ER-T2 mice for sequential mutagenesis" was retracted in 2016. Reasons: errors in the results or conclusions; unreliable results or conclusions.

To examine the leakiness of Cre-ER^T2^ in *Col1a1^FRT-STOP-FRT-Cre-ER-T2^* mice, tissues from 6-month-old *Col1a1^FRT-STOP-FRT-Cre-ER-T2^; Rosa26^mTmG/+^* mice were examined by immunofluorescence with (*n*=2) and without (*n*=2) tamoxifen treatment (Fig. 6). In the absence of tamoxifen, there was widespread tdTomato expression without evidence of eGFP expression in any of the tissues examined (Fig. 6A). When tissues were collected 30 days after intraperitoneal delivery of one dose of 75 mg tamoxifen/kg body weight in corn oil, there continued to be widespread tdTomato expression without evidence of eGFP expression in any of the tissues examined (Fig. 6B). These results indicate that the STOP cassette is functional and does not allow for Cre-ER^T2^-mediated transcription in the absence of Flp-mediated recombination and excision of the STOP cassette.

**Fig. 6.** **Characterization of *Col1a1^FRT-STOP-FRT-Cre-ER-T2^* mice.** (A) Immunofluorescence of tissues from 6-month-old *Col1a1^FRT-STOP-FRT-Cre-ER-T2^; Rosa26^mTmG/+^* mice (*n*=2) without tamoxifen treatment show widespread tdTomato expression and no eGFP expression. (B) Immunofluorescence of tissues collected 30 days after one dose of intraperitoneal tamoxifen in 6-month-old mice (*n*=2) continue to show widespread tdTomato expression and no eGFP expression, indicating that the STOP cassette prevents expression of Cre-ER^T2^ in the absence of FlpO-mediated recombination and excision of the STOP cassette. Scale bars: 50 µm.

To determine whether the STOP cassette for the *Col1a1^FRT-STOP-FRT-Cre-ER-T2^* allele can be excised by Flp-mediated recombination *in vivo*, mice with the *Col1a1^FRT-STOP-FRT-Cre-ER-T2^* allele were crossed to *Kras^FRT-STOP-FRT-G12D/+^; p53^FRT/FRT^* mice (Lee et al., 2012) to generate *Col1a1^FRT-STOP-FRT-Cre-ER-T2/+^; Kras^FRT-STOP-FRT-G12D/+^; p53^FRT/FRT^* mice. Adenovirus expressing mammalian optimized Flp recombinase (Adeno-FlpO) was injected into the hindlimb of these mice to generate primary soft-tissue sarcomas. Once sarcomas developed, the bulk tumor tissues were excised and dissociated into single-cell suspensions and cultured *in vitro*. Genomic DNA was isolated from these cells and the recombination of the STOP cassette was verified by PCR (Fig. 7A). Tail DNA taken at the time of genotyping from a *Col1a1^FRT-Cre-ER-T2-FRT^* mouse was used as a positive control for the absence of STOP cassette, and tail DNA taken at the time of genotyping from a *Col1a1^FRT-STOP-FRT-Cre-ER-T2^* mouse was used as a negative control for the recombined STOP cassette.

The article "The generation and characterization of novel Col1a1FRT-Cre-ER-T2-FRT and Col1a1FRT-STOP-FRT-Cre-ER-T2 mice for sequential mutagenesis" was retracted in 2016. Reasons: errors in the results or conclusions; unreliable results or conclusions.

**Fig. 7.** **Characterization of primary sarcomas generated in *Col1a1^FRT-STOP-FRT-Cre-ER-T2^; Kras^FRT-STOP-FRT-G12D/+^; p53^FRT/FRT^; Rosa26^mTmG/+^* mice.** Primary sarcomas were generated by intramuscular injection of adenovirus expressing FlpO recombinase into the hindlimb of 6-week-old *Col1a1^FRT-STOP-FRT-Cre-ER-T2^; Kras^FRT-STOP-FRT-G12D/+^; p53^FRT/FRT^; Rosa26^mTmG/+^* mice. (A) Primary sarcoma cells were isolated by dissociation of the bulk tumor and subsequent *in vitro* passage. The excision of the STOP cassette in the *Col1a1^FRT-STOP-FRT-Cre-ER-T2^* allele was confirmed via PCR for two tumors using primers FWD4 and REV2. Tail DNA from untreated *Col1a1^FRT-Cre-ER-T2-FRT^* mice serves as positive control for the absence of the STOP cassette, whereas the tail DNA from *Col1a1^FRT-STOP-FRT-Cre-ER-T2^* mice serves as negative control for the retention of the STOP cassette. (B) After tumor formation in *Col1a1^FRT-STOP-FRT-Cre-ER-T2^; Kras^FRT-STOP-FRT-G12D/+^; p53^FRT/FRT^; Rosa26^mTmG/+^* mice (*n*=2), one dose of tamoxifen was delivered by intraperitoneal injection. Tumors were collected 10 days after tamoxifen delivery. Immunofluorescence of tumor tissue showed no eGFP expression (iii), with the whole tumor retaining tdTomato (iv). (C) After tumor formation in *Col1a1^FRT-STOP-FRT-Cre-ER-T2^; Kras^FRT-STOP-FRT-G12D/+^; p53^FRT/FRT^; Rosa26^mTmG/+^* mice (*n*=2), 4-hydroxytamoxifen was delivered by intramuscular injection at the site of the tumor. Tumors were collected 10 days after 4-hydroxytamoxifen delivery. Immunofluorescence of tumor tissue showed scattered tdTomato expression labeling tumor vasculature and other stromal cells (iv), with the majority of tumor tissue expressing eGFP, which labels tumor parenchyma (iii). (D) After tumor formation in *Col1a1^FRT-STOP-FRT-Cre-ER-T2^; Kras^FRT-STOP-FRT-G12D/+^; p53^FRT/FRT^; Rosa26^mTmG/+^* mice (*n*=2), one dose of 4-hydroxytamoxifen was delivered by subcutaneous injection between the scapula. Tumors were collected 24 h after 4-hydroxytamoxifen delivery. Immunofluorescence of tumor tissue showed widespread tdTomato expression (iv), with small clusters of cells expressing eGFP, which labels tumor parenchyma (iii). (E) After tumor formation in *Col1a1^FRT-STOP-FRT-Cre-ER-T2^; Kras^FRT-STOP-FRT-G12D/+^; p53^FRT/FRT^; Rosa26^mTmG/+^* mice (*n*=1), 4-hydroxytamoxifen was delivered by one dose of intraperitoneal injection, followed by three doses of subcutaneous injection between the scapula. Doses of 4-hydroxytamoxifen were given in 24 h intervals. Tumors were collected 1 day after the last dose of 4-hydroxytamoxifen delivery. Immunofluorescence of tumor tissue showed scattered tdTomato expression labeling tumor vasculature and other stromal cells (iv), and cells with varying degrees of eGFP expression (iii). These results indicate that the *Col1a1^FRT-STOP-FRT-Cre-ER-T2^* is functional and can be utilized for sequential mutagenesis *in vivo*. Scale bars: 100 µm.

The article "The generation and characterization of novel Col1a1FRT-Cre-ER-T2-FRT and Col1a1FRT-STOP-FRT-Cre-ER-T2 mice for sequential mutagenesis" was retracted in 2016. Reasons: errors in the results or conclusions; unreliable results or conclusions.

To examine the functionality of the *Col1a1^FRT-STOP-FRT-Cre-ER-T2^* allele in a tumor model, these mice were crossed to *Kras^FRT-STOP-FRT-G12D/+^; p53^FRT/FRT^; Rosa26^mTmG/+^* mice to generate *Col1a1^FRT-STOP-FRT-Cre-ER-T2^; Kras^FRT-STOP-FRT-G12D/+^; p53^FRT/FRT^; Rosa26^mTmG/+^* mice. Primary sarcomas were generated in the hindlimb of these mice by intramuscular injection of Adeno-FlpO. After the initial tumor was palpated in the *Col1a1^FRT-STOP-FRT-Cre-ER-T2^; Kras^FRT-STOP-FRT-G12D/+^; p53^FRT/FRT^; Rosa26^mTmG/+^* mice, a single dose of 75 mg tamoxifen/kg body weight in corn oil was delivered via intraperitoneal injection. Tumors (*n*=2) were collected 10 days after the tamoxifen delivery, and immunofluorescence was used to evaluate tdTomato and eGFP expression (Fig. 7B). Unexpectedly, the whole tumor tissue remained tdTomato-positive without any evidence of eGFP expression. Because the STOP cassette can be appropriately removed by FlpO, as shown in Fig. 7A, the lack of tdTomato deletion and eGFP expression might be due to inadequate levels and/or penetration of the active tamoxifen metabolite into the tumor tissue. Therefore, alternative approaches of tamoxifen delivery were explored in subsequent cohorts. After the initial tumor was palpated in a second cohort (*n*=2) of *Col1a1^FRT-STOP-FRT-Cre-ER-T2^; Kras^FRT-STOP-FRT-G12D/+^; p53^FRT/FRT^; Rosa26^mTmG/+^* mice, a single dose of 0.75 mg 4-hydroxytamoxifen in DMSO was delivered via intratumoral injection. Tumors were collected 10 days after the 4-hydroxytamoxifen delivery, and tdTomato and eGFP expression were evaluated by immunofluorescence (Fig. 7C). In contrast to tumors from mice that were given intraperitoneal tamoxifen injection, the bulk tumor from mice that received intratumoral 4-hydroxytamoxifen were mostly eGFP-positive with scattered tdTomato expression. For another set (*n*=2) of *Col1a1^FRT-STOP-FRT-Cre-ER-T2^; Kras^FRT-STOP-FRT-G12D/+^; p53^FRT/FRT^; Rosa26^mTmG/+^*mice, a single dose of 2 mg 4-hydroxytamoxifen in PBS was delivered via subcutaneous injection between the scapula. Twenty-four hours following the single injection, the tumors were harvested, and tdTomato and eGFP expression were evaluated by immunofluorescence (Fig. 7D). These tumors demonstrated areas of small clusters of cells that were eGFP-positive, although the majority of the tumors remained tdTomato-positive. This demonstrates that a single high dose of 4-hydroxytamoxifen delivered systemically can penetrate the bulk tumor, but only to a limited area that is likely well perfused. Finally, after the initial tumor was palpated in the lower limb in a *Col1a1^FRT-STOP-FRT-Cre-ER-T2^; Kras^FRT-STOP-FRT-G12D/+^; p53^FRT/FRT^; Rosa26^mTmG/+^* mouse, one dose of 2 mg 4-hydroxytamoxifen in PBS was delivered via intraperitoneal injection. Twenty-four hours following the first injection, 2 mg of 4-hydroxytamoxifen in PBS was delivered via subcutaneous injection between the scapula. Two more subcutaneous injections of 4-hydroxytamoxifen were delivered at the same site every 24 h for a total of four doses (one intraperitoneal and three subcutaneous). This tumor was collected 1 day after the last dose of 4-hydroxytamoxifen, and tdTomato and eGFP expression were evaluated by immunofluorescence (Fig. 7E). This tumor demonstrated scattered areas with high eGFP expression and larger areas with diffusely lower eGFP expression, and scattered tdTomato expression. This suggests that administration of multiple high doses of systemic 4-hydroxytamoxifen is capable of penetrating the tumor tissue to enable Cre-ER^T2^-mediated recombination of *loxP* sites.

The article "The generation and characterization of novel Col1a1FRT-Cre-ER-T2-FRT and Col1a1FRT-STOP-FRT-Cre-ER-T2 mice for sequential mutagenesis" was retracted in 2016. Reasons: errors in the results or conclusions; unreliable results or conclusions.

Taken together, these results show that the Cre-ER^T2^ in both *Col1a1^FRT-Cre-ER-T2-FRT^* and *Col1a1^FRT-STOP-FRT-Cre-ER-T2^* mice is functional and that the recombinase activity in both mice can be potently induced by the active tamoxifen metabolite. Additionally, the expression of Cre-ER^T2^ in *Col1a1^FRT-STOP-FRT-Cre-ER-T2^* mice is tightly controlled by the STOP cassette. However, in this primary sarcoma model, penetration of the active tamoxifen metabolite into the tumor following a single intraperitoneal tamoxifen injection is insufficient to activate the *Col1a1^FRT-STOP-FRT-Cre-ER-T2^* allele. The limited penetration of the active tamoxifen metabolite after a single intraperitoneal injection of tamoxifen might be due to the large size (approximately 200 mm^3^) of the sarcomas at the time of palpation and thus might not be a limitation for other tumor models in which the tumors are smaller. Even in the primary sarcoma model, the limited penetration following a single intraperitoneal injection of tamoxifen can be overcome by several doses of 4-hydroxytamoxifen delivered by intraperitoneal and subcutaneous routes. Finally, in the *Col1a1^FRT-Cre-ER-T2-FRT^* mice there is a time-dependent recombinase activity of Cre-ER^T2^ in the absence of tamoxifen exposure, which might limit its utility in certain tissues for experiments that would require waiting several months before the administration of tamoxifen.

The article "The generation and characterization of novel Col1a1FRT-Cre-ER-T2-FRT and Col1a1FRT-STOP-FRT-Cre-ER-T2 mice for sequential mutagenesis" was retracted in 2016. Reasons: errors in the results or conclusions; unreliable results or conclusions.

## DISCUSSION

The primary mouse model is an important tool to study biological processes *in vivo*; therefore, novel mouse strains and mouse models provide an opportunity for scientific advancement. Here, we have generated two novel mouse strains to facilitate more precise manipulation of the mouse genome to answer complex questions.

The two novel mouse strains take advantage of different site-specific recombinase systems to enable sequential mutagenesis separated in time and cellular location. These novel mouse strains will facilitate the study of complex questions in development, normal tissue homeostasis and disease processes, such as cancer. For example, these strains have a number of advantages for studying the role of genes in either tumor cells or stroma. First, the knock-in alleles of both novel mouse strains are targeted to the ubiquitously expressed *Col1a1* locus instead of the frequently used *Rosa26* locus. This *Col1a1* site was selected with the available *Rosa26* knock-in alleles in mind*.* An advantage of knock-in alleles over other transgenic approaches that generate alleles by random integration into the mouse genome is that the precise location of the knock-in allele is known. However, each mouse can only harbor two different copies of a mutant gene at one locus. Because there are many *Rosa26* knock-in alleles, ranging from mutant genes to fluorescent reporters, the placement of the two novel Flp-regulated Cre-ER^T2^ alleles at the *Col1a1* locus retains the availability of both alleles of the *Rosa26* locus for other genes of interest.

Our results indicate that the *Col1a1* locus is a good alternative to the *Rosa26* locus for ubiquitous gene expression, as noted by diffuse eGFP expression after tamoxifen-mediated deletion of tdTomato in *Col1a1^FRT-Cre-ER-T2-FRT^; Rosa26^mTmG/+^* mice. In addition, Cre-ER^T2^ is tightly regulated by the STOP cassette in *Col1a1^FRT-STOP-FRT-Cre-ER-T2^; Rosa26^mTmG/+^* mice and, after successful removal of the STOP cassette by Adeno-FlpO, Cre-ER^T2^ can be efficiently activated by 4-hydroxytamoxifen in primary soft-tissue sarcomas via intratumoral injection or multiple systemic injections to express eGFP in the tumor parenchyma.

A limitation of the *Col1a1^FRT-Cre-ER-T2-FRT^* mice is the age-dependent tissue-specific Cre-ER^T2^ activity independent of exogenous tamoxifen administration, which is most pronounced in the pancreas and the liver. This could result from a number of factors, including tissue-specific basal expression from the *Col1a1* locus, tissue-specific exposure to endogenous estrogens that might activate Cre-ER^T2^, and the rate of tissue-specific protein turnover. Tissues that are less affected include the bone marrow and the brain. This might limit the scope of experiments that can be performed with the *Col1a1^FRT-Cre-ER-T2-FRT^* allele to younger mice, to a shorter timeframe for sequential mutagenesis, and/or to specific organs, especially in older mice. In contrast, we did not observe any leakiness from Cre-ER^T2^ in the *Col1a1^FRT-STOP-FRT-Cre-ER-T2^* mice. Thus, the age of mice for experiments with this allele does not seem to be a critical experimental variable. In primary sarcomas initiated by Adeno-FlpO from *Col1a1^FRT-STOP-FRT-Cre-ER-T2^; Kras^FRT-STOP-FRT-G12D/+^; p53^FRT/FRT^; Rosa26^mTmG/+^* mice, we were able to activate Cre-ER^T2^ in tumor cells by intratumoral administration of 4-hydroxytamoxifen or multiple doses of systemic 4-hydroxytamoxifen. However, experiments with intraperitoneal injection of a single dose of tamoxifen failed to activate Cre-ER^T2^ in primary sarcomas when they were approximately 200 mm^3^. Therefore, the delivery of an adequate level of active tamoxifen metabolites into the tumor will be necessary to apply this system in established sarcomas. In addition to injecting 4-hydroxytamoxifen into the tumor or systemically, another approach that could be utilized is delivery of tamoxifen in the food (Schönhuber et al., 2014).

The article "The generation and characterization of novel Col1a1FRT-Cre-ER-T2-FRT and Col1a1FRT-STOP-FRT-Cre-ER-T2 mice for sequential mutagenesis" was retracted in 2016. Reasons: errors in the results or conclusions; unreliable results or conclusions.

Recently, *in vivo* manipulations of the mouse genome have been achieved using the CRISPR/Cas9 system to generate tumors, for example in the liver and lung, via: hydrodynamic injections (Xue et al., 2014), adenoviral delivery of both sgRNA and Cas9 (Sánchez-Rivera et al., 2014), or adenoviral delivery of sgRNA and Cre into *Rosa26^loxP-STOP-loxP-Cas9^* mice (Platt et al., 2014). There are distinct advantages and disadvantages to using either the CRISPR/Cas9 or the Cre-*loxP* recombinase systems to model cancer depending on the application. For example, the CRISPR/Cas9 system does not require the generation of mice with multiple mutant alleles. Therefore, the CRISPR/Cas9 system enables testing of the impact of different gene mutations on a cancer model more quickly. However, the Cre-*loxP* recombinase system can be much more efficient in generating a specific gene mutation. One exciting application of the CRISPR/Cas9 system would be to combine the time efficiency of the CRISPR/Cas9 system with the spatial and temporal control of stepwise genomic manipulations with the Flp-*FRT*-mediated Cre-ER^T2^ mouse strains. Specifically, the *Col1a1^FRT-STOP-FRT-Cre-ER-T2^* mouse strain could be used in combination with *Rosa26^loxP-STOP-loxP-Cas9^* mice such that *in vivo* genome-scale screening would be possible to evaluate cooperating mutations for cancer initiation and maintenance.

The article "The generation and characterization of novel Col1a1FRT-Cre-ER-T2-FRT and Col1a1FRT-STOP-FRT-Cre-ER-T2 mice for sequential mutagenesis" was retracted in 2016. Reasons: errors in the results or conclusions; unreliable results or conclusions.

In summary, we have generated two complementary novel Flp-*FRT*-regulated Cre-ER^T2^ mouse strains that can be used for sequential mutagenesis with the Flp-*FRT* and the Cre-*loxP* systems. The *Col1a1^FRT-Cre-ER-T2-FRT^* allele can be combined with FlpO, *FRT*-flanked, and *loxP*-regulated genes to generate mice where distinct mutations can be expressed in neighboring cells to study intercellular communications such as those between tumor parenchymal and stromal cells. Furthermore, the *Col1a1^FRT-STOP-FRT-Cre-ER-T2^* allele can be combined with FlpO, *FRT*-flanked and *loxP-*regulated genes to generate mice in which two distinct mutations can be expressed in a single cell sequentially. We anticipate that this allele will provide a tightly regulated tool to study sequential mutagenesis in cancer development and to test the role of genes in tumor maintenance by mimicking therapeutic target inhibition or activation during cancer therapy.

## MATERIALS AND METHODS

All animal experiments were performed according to protocols approved by the Duke University Institutional Animal Care and Use Committee.

### Generation of novel mouse models

Knock-in alleles *Col1a1^FRT- Cre-ER-T2-FRT^* and *Col1a1^FRT-STOP-FRT- Cre-ER-T2^* were generated by targeting the *FRT-Cre-ER^T2^-FRT-NEO* or the *FRT-STOP*-*FRT-Cre-ER^T2^-NEO* constructs to the *Col1a1* locus in 129/SVJae embryonic stem cells (ES cells). 129/SVJae ES cells were selected in neomycin (G418), and screened for homologous recombination at the *Col1a1* locus by PCR and Southern blot. ES cells that were successfully targeted at the *Col1a1* locus were injected into C57BL/6 blastocysts, which were then implanted into pseudo-pregnant mice. Male chimeras were bred to female C57BL/6 mice and the resulting progeny with brown-colored coat (i.e. 129/SVJae-derived) were analyzed for germline transmission of the targeted alleles. Mice with germline transmission were crossed to the *Rosa26^PhiC31^* (Raymond and Soriano, 2007), which removed the *attB/attP*-flanked neomycin cassette.

### Adenovirus-mediated sarcomagenesis

Mouse models of soft-tissue sarcoma were generated in a mixed 129/SVJae and C57BL/6 background using a combination of previously described alleles: *Kras^FRT-STOP-FRT-G12D^* (Young et al., 2011), *p53^FRT^* (Lee et al., 2012) and *Rosa26^mTmG^* (Muzumdar et al., 2007). A working solution of replication-deficient adenovirus expressing FlpO recombinase (Adeno-FlpO) was generated by precipitating 25 µl of Adeno-FlpO stock (University of Iowa Gene Transfer Vector Core, Iowa City, IA) with 3 µl 2 M CaCl_2_ (Sigma-Aldrich, St Louis, MO) and 600 µl MEM (Sigma-Aldrich, St Louis, MO) as previously described (Kirsch et al., 2007). The working solution was then incubated at room temperature for 15 min prior to use. Soft-tissue sarcomas in the mouse hindlimb were generated by intramuscular (IM) injection of 50 µl Adeno-FlpO working solution via a 28.5-gauge insulin syringe (BD Biosciences, Franklin Lakes, NJ).

The article "The generation and characterization of novel Col1a1FRT-Cre-ER-T2-FRT and Col1a1FRT-STOP-FRT-Cre-ER-T2 mice for sequential mutagenesis" was retracted in 2016. Reasons: errors in the results or conclusions; unreliable results or conclusions.

### 4-hydroxytamoxifen and tamoxifen injections

(Z)-4-hydroxytamoxifen (Sigma-Aldrich, St Louis, MO), or 4-OHT, was first dissolved in 100% ethanol at a concentration of 250 mg/ml, and then diluted with dimethyl sulfoxide (DMSO) (Sigma-Aldrich, St Louis, MO) to a final working solution concentration of 25 mg/ml. Soft-tissue sarcoma in the mouse hindlimb was then infiltrated with a single intratumoral injection of 30 µl 4-OHT (0.75 mg) working solution via a 28.5-gauge insulin syringe. Alternatively, 4-OHT was dissolved in one-to-one ratio of 100% ethanol and Kolliphor^®^ EL (Sigma-Aldrich, St Louis, MO) at 20 mg/ml, and then diluted with PBS to 10 mg/ml. Mice were treated with either 200 µl intraperitoneal or subcutaneous injections of 4-OHT via a 27.5-gauge insulin syringe. Tamoxifen (Sigma-Aldrich, St Louis, MO) was first dissolved in corn oil (Sigma-Aldrich, St Louis, MO) at a concentration of 20 mg/ml. Mice were treated with a single intraperitoneal injection of tamoxifen at 75 mg/kg body weight via a 27.5-gauge insulin syringe.

### Tumor cell isolation and culture

Sarcomas were removed after animals were sacrificed and the tumors were digested with tissue digestion buffer consisting of 5 mg/ml collagenase IV (Sigma-Aldrich, St Louis, MO), 2.5 U/ml dispase (BD Biosciences, Franklin Lakes, NJ) and 0.05% trypsin (Life Technologies, Carlsbad, CA) at 37°C for 40 min. The resulting mixture was strained through a 70-µm filter (BD Biosciences, Franklin Lakes, NJ), and filtered cells were re-suspended in culture medium consisting of DMEM/F12 (Life Technologies, Carlsbad, CA) with 10% fetal bovine serum (Sigma-Aldrich, St Louis, MO) and 1× penicillin/streptomycin (Life Technologies, Carlsbad, CA).

### Polymerase chain reactions

DNA was isolated using the DNeasy Blood and Tissue Kit (Qiagen, Venlo, Limburg) and PCR experiments were performed with a C1000 Touch Thermal Cycler (Bio-Rad, Hercules, CA). Nucleic acid concentrations were measured using NanoDrop 1000 (Thermo Scientific, Waltham, MA). The location of the primer sequences relative to the targeted alleles are shown in Fig. 3 and the sequences are as follows: 5′-GGGCTCGACGACTAGGTTAA-3′ (FWD1), 5′-GAGATCTGGGAATGAAGTACGTG-3′ (FWD2), 5′-ATCATGTCTGGATCCCCATC-3′ (FWD3), 5′-GCAACGTGCTGGTTATTGTG-3′ (FWD4), 5′-GCCTGTCTTATGCCTTAGACC-3′ (REV1), 5′-CCAGCATCCACATTCTCCTT-3′ (REV2). FWD1 and REV1 amplify a 395-bp product for *Col1a1^FRT-Cre-ER-T2-FRT^* and a 360-bp product for *Col1a1^FRT-STOP-FRT-Cre-ER-T2^*. FWD2 and REV1 amplify a 156-bp product for the wild-type *Col1a1* locus. FWD3 and REV2 amplify a 479-bp product if the STOP cassette is not excised for *Col1a1^FRT-STOP-FRT-Cre-ER-T2^*. FWD4 and REV2 amplify a 489-bp product for *Col1a1^FRT-Cre-ER-T2-FRT^*, or if the STOP cassette is excised for *Col1a1^FRT-STOP-FRT-Cre-ER-T2^*. FWD4 and REV1 amplify a 435-bp product for *Col1a1^FRT-Cre-ER-T2-FRT^* if the Cre-ER^T2^ cassette is excised.

The article "The generation and characterization of novel Col1a1FRT-Cre-ER-T2-FRT and Col1a1FRT-STOP-FRT-Cre-ER-T2 mice for sequential mutagenesis" was retracted in 2016. Reasons: errors in the results or conclusions; unreliable results or conclusions.

PCR for the NEO cassette amplifies a 540-bp product if the NEO cassette is present in the *Col1a1^FRT-Cre-ER-T2-FRT-NEO^* and *Col1a1^FRT-STOP-FRT-Cre-ER-T2-NEO^* mice using the following two primers: 5′-CCTCGTGCTTTACGGTATCGCC-3′ (FWD5), 5′-GCCTGTCTTATGCCTTAGACC-3′ (REV1). The *Rosa26^PhiC31^* PCR was performed using primers as previously described (Raymond and Soriano, 2007).

One touchdown PCR program was used for all reactions: (1) melting at 94°C for 180 s; (2) for 15 cycles, melting at 94°C for 45 s, annealing at 64°C for 45 s with −0.5°C per cycle, elongating at 72°C for 60 s; (3) for 25 cycles, melting at 94°C for 45 s, annealing at 57°C for 45 s, elongating at 72°C for 60 s; (4) elongating at 72°C for 600 s.

### Frozen sectioning and immunofluorescence

For frozen sectioning, tumor and tissue specimens were dissected, embedded in OCT (Tissue-Tek, Torrance, CA) and frozen over dry ice. Frozen specimens and 10-µm sections generated via a cryostat (Leica Microsystems, Wetzlar, Germany) were stored unfixed at −80°C. For immunofluorescence, slides were incubated with Alexa-Fluor-488-conjugated rabbit anti-GFP antibody (Life Technologies, Carlsbad, CA) at a concentration of 1:500 for 1 h at room temperature. Slides were then counterstained with 4′,6-diamidino-2-phenylindole (DAPI) (Sigma-Aldrich, St Louis, MO). Images were captured with a DM5500B microscope (Leica Microsystems, Wetzlar, Germany) using Leica Application Suite software.

### Resource sharing

The *Col1a1^FRT-Cre-ER-T2-FRT^* and *Col1a1^FRT-STOP-FRT-Cre-ER-T2^* mouse strains in the mixed C57BL/6 and 129/SVJae background will be available at The Jackson Laboratory Repository with the JAX Stock Nos. 027750 and 027751. The strains are also available upon written request to D.G.K.

## References

[DMM021204C1] BlumJ. M., AñóL., LiZ., Van MaterD., BennettB. D., SachdevaM., LagutinaI., ZhangM., MitoJ. K., DoddL. G.et al. (2013). Distinct and overlapping sarcoma subtypes initiated from muscle stem and progenitor cells. *Cell Rep.* 5, 933-940. 10.1016/j.celrep.2013.10.02024239359PMC3893104

[DMM021204C2] DymeckiS. M. (1996). Flp recombinase promotes site-specific DNA recombination in embryonic stem cells and transgenic mice. *Proc. Natl. Acad. Sci. USA* 93, 6191-6196. 10.1073/pnas.93.12.61918650242PMC39212

[DMM021204C3] El MarjouF., JanssenK.-P., ChangB. H.-J., LiM., HindieV., ChanL., LouvardD., ChambonP., MetzgerD. and RobineS. (2004). Tissue-specific and inducible Cre-mediated recombination in the gut epithelium. *Genesis* 39, 186-193. 10.1002/gene.2004215282745

[DMM021204C4] HaigisK. M., KendallK. R., WangY., CheungA., HaigisM. C., GlickmanJ. N., Niwa-KawakitaM., Sweet-CorderoA., Sebolt-LeopoldJ., ShannonK. M.et al. (2008). Differential effects of oncogenic K-Ras and N-Ras on proliferation, differentiation and tumor progression in the colon. *Nat. Genet.* 40, 600-608. 10.1038/ng.11518372904PMC2410301

[DMM021204C5] IndraA. K., WarotX., BrocardJ., BornertJ.-M., XiaoJ.-H., ChambonP. and MetzgerD. (1999). Temporally-controlled site-specific mutagenesis in the basal layer of the epidermis: comparison of the recombinase activity of the tamoxifen-inducible Cre-ER(T) and Cre-ER(T2) recombinases. *Nucleic Acids Res.* 27, 4324-4327. 10.1093/nar/27.22.432410536138PMC148712

[DMM021204C6] JacksonE. L., WillisN., MercerK., BronsonR. T., CrowleyD., MontoyaR., JacksT. and TuvesonD. A. (2001). Analysis of lung tumor initiation and progression using conditional expression of oncogenic K-ras. *Genes Dev.* 15, 3243-3248. 10.1101/gad.94300111751630PMC312845

[DMM021204C7] KirschD. G., DinulescuD. M., MillerJ. B., GrimmJ., SantiagoP. M., YoungN. P., NielsenG. P., QuadeB. J., ChaberC. J., SchultzC. P.et al. (2007). A spatially and temporally restricted mouse model of soft tissue sarcoma. *Nat. Med.* 13, 992-997. 10.1038/nm160217676052

[DMM021204C8] LeeC.-L., ModingE. J., HuangX., LiY., WoodliefL. Z., RodriguesR. C., MaY. and KirschD. G. (2012). Generation of primary tumors with Flp recombinase in FRT-flanked p53 mice. *Dis. Model. Mech.* 5, 397-402. 10.1242/dmm.00908422228755PMC3339833

[DMM021204C9] MarinoS., VooijsM., van Der GuldenH., JonkersJ. and BernsA. (2000). Induction of medulloblastomas in p53-null mutant mice by somatic inactivation of Rb in the external granular layer cells of the cerebellum. *Genes Dev.* 14, 994-1004.10783170PMC316543

[DMM021204C10] MeuwissenR., LinnS. C., LinnoilaR. I., ZevenhovenJ., MooiW. J. and BernsA. (2003). Induction of small cell lung cancer by somatic inactivation of both Trp53 and Rb1 in a conditional mouse model. *Cancer Cell* 4, 181-189. 10.1016/S1535-6108(03)00220-414522252

[DMM021204C11] ModingE. J., LeeC.-L., CastleK. D., OhP., MaoL., ZhaS., MinH. D., MaY., DasS. and KirschD. G. (2014). Atm deletion with dual recombinase technology preferentially radiosensitizes tumor endothelium. *J. Clin. Invest.* 124, 3325-3338. 10.1172/JCI7393225036710PMC4109553

[DMM021204C12] ModingE. J., CastleK. D., PerezB. A., OhP., MinH. D., NorrisH., MaY., CardonaD. M., LeeC.-L. and KirschD. G. (2015). Tumor cells, but not endothelial cells, mediate eradication of primary sarcomas by stereotactic body radiation therapy. *Sci. Transl. Med.* 7, 278ra34 10.1126/scitranslmed.aaa4214PMC436013525761890

[DMM021204C13] MuzumdarM. D., TasicB., MiyamichiK., LiL. and LuoL. (2007). A global double-fluorescent Cre reporter mouse. *Genesis* 45, 593-605. 10.1002/dvg.2033517868096

[DMM021204C14] O'GormanS., FoxD. T. and WahlG. M. (1991). Recombinase-mediated gene activation and site-specific integration in mammalian cells. *Science* 251, 1351-1355. 10.1126/science.19006421900642

[DMM021204C15] OrbanP. C., ChuiD. and MarthJ. D. (1992). Tissue- and site-specific DNA recombination in transgenic mice. *Proc. Natl. Acad. Sci. USA* 89, 6861-6865. 10.1073/pnas.89.15.68611495975PMC49604

[DMM021204C16] PlattR. J., ChenS., ZhouY., YimM. J., SwiechL., KemptonH. R., DahlmanJ. E., ParnasO., EisenhaureT. M., JovanovicM.et al. (2014). CRISPR-Cas9 knockin mice for genome editing and cancer modeling. *Cell* 159, 440-455. 10.1016/j.cell.2014.09.01425263330PMC4265475

[DMM021204C17] RaymondC. S. and SorianoP. (2007). High-efficiency FLP and PhiC31 site-specific recombination in mammalian cells. *PLoS ONE* 2, e162 10.1371/journal.pone.000016217225864PMC1764711

[DMM021204C18] SaamJ. R. and GordonJ. I. (1999). Inducible gene knockouts in the small intestinal and colonic epithelium. *J. Biol. Chem.* 274, 38071-38082. 10.1074/jbc.274.53.3807110608876

[DMM021204C19] Sánchez-RiveraF. J., PapagiannakopoulosT., RomeroR., TammelaT., BauerM. R., BhutkarA., JoshiN. S., SubbarajL., BronsonR. T., XueW.et al. (2014). Rapid modelling of cooperating genetic events in cancer through somatic genome editing. *Nature* 516, 428-431. 10.1038/nature1390625337879PMC4292871

[DMM021204C20] SauerB. and HendersonN. (1988). Site-specific DNA recombination in mammalian cells by the Cre recombinase of bacteriophage P1. *Proc. Natl. Acad. Sci. USA* 85, 5166-5170. 10.1073/pnas.85.14.51662839833PMC281709

[DMM021204C21] SchönhuberN., SeidlerB., SchuckK., VeltkampC., SchachtlerC., ZukowskaM., EserS., FeyerabendT. B., PaulM. C., EserP.et al. (2014). A next-generation dual-recombinase system for time- and host-specific targeting of pancreatic cancer. *Nat. Med.* 20, 1340-1347. 10.1038/nm.364625326799PMC4270133

[DMM021204C22] ShaiA., DankortD., JuanJ., GreenS. and McMahonM. (2015). TP53 silencing bypasses growth arrest of BRAFV600E-induced lung tumor cells in a two-switch model of lung tumorigenesis. *Cancer Res.* 10.1158/0008-5472.CAN-14-3701.PMC452643026001956

[DMM021204C23] SutherlandK. D., ProostN., BrounsI., AdriaensenD., SongJ.-Y. and BernsA. (2011). Cell of origin of small cell lung cancer: inactivation of Trp53 and Rb1 in distinct cell types of adult mouse lung. *Cancer Cell* 19, 754-764. 10.1016/j.ccr.2011.04.01921665149

[DMM021204C24] SutherlandK. D., SongJ.-Y., KwonM. C., ProostN., ZevenhovenJ. and BernsA. (2014). Multiple cells-of-origin of mutant K-Ras-induced mouse lung adenocarcinoma. *Proc. Natl. Acad. Sci. USA* 111, 4952-4957. 10.1073/pnas.131996311124586047PMC3977239

[DMM021204C25] WangY., KrushelL. A. and EdelmanG. M. (1996). Targeted DNA recombination in vivo using an adenovirus carrying the cre recombinase gene. *Proc. Natl. Acad. Sci. USA* 93, 3932-3936. 10.1073/pnas.93.9.39328632992PMC39462

[DMM021204C26] XueW., ChenS., YinH., TammelaT., PapagiannakopoulosT., JoshiN. S., CaiW., YangG., BronsonR., CrowleyD. G.et al. (2014). CRISPR-mediated direct mutation of cancer genes in the mouse liver. *Nature* 514, 380-384. 10.1038/nature1358925119044PMC4199937

[DMM021204C27] YoungN. P., CrowleyD. and JacksT. (2011). Uncoupling cancer mutations reveals critical timing of p53 loss in sarcomagenesis. *Cancer Res.* 71, 4040-4047. 10.1158/0008-5472.CAN-10-456321512139PMC3160277

